The article "3D Garment Design Model Based on Convolution Neural Network and Virtual Reality" was published in 2022. Journal: Comput Intell Neurosci.

# 3D Garment Design Model Based on Convolution Neural Network and Virtual Reality

**DOI:** 10.1155/2022/9187244

**Published:** 2022-06-27

**Authors:** Liu Fengyi, Siru Liu

**Affiliations:** Lu Xun Academy of Fine Arts, Liaoning, Dalian 116021, China

## Abstract

The development of virtual reality technology has promoted the unceasing reform and development in the field of fashion design. Aiming at the key technologies and research difficulties in 3D clothing design, the structure of convolution neural network was designed, and a 3D clothing design model based on convolution neural network and virtual reality was constructed. By designing experiments, the average error, matching rate, prediction accuracy, pressure value, and other evaluation indexes are used to measure the performance of convolution neural network model in virtual reality three-dimensional clothing design. The results show that: first, the convolution neural network has the fastest training speed, with the maximum error of 1.63% and the average error of 0.48%. Second, with the increase of parameters, the matching degree of each part of the version and the corresponding data of the human body will gradually increase, the matching rate will slowly improve, and finally tends to 0.9 or so to achieve stability, Thirdly, the prediction accuracy of the convolution neural network is 92.689%, and the loss value is the least. Fourthly, in the virtual fitting and garment wearing experiments, the fit of the sample is within the allowed range, indicating that the automatic generation of fit sample has wearability and rationality.

## 1. Introduction 

Clothing is an important part of human society and culture and an important manifestation of human spiritual civilization [1]. With the improvement of people's material living conditions, consumers' pursuit of clothing styles and fabrics has changed, and they are increasingly pursuing personalized clothing design. The traditional two-dimensional fashion design method cannot meet the requirements of high efficiency and low cost of product development of garment enterprises and cannot adapt to the fashion pursuit of consumers. With the rapid development of computer science and technology and the continuous innovation of the garment industry, the garment design is gradually expanding from the functions of placing codes, arranging materials and style design based on two-dimensional graphics to the functions of three-dimensional virtual body scanning, virtual design, virtual fitting, and virtual display. In the design of the clothing, by means of the real-time interaction provided by the new information technology of virtual reality, the original pure two-dimensional design method is gradually transformed into a three-dimensional design visible on the computer. The three-dimensional design fully reflects the three-dimensional integration of human beings in this environment by constructing dummy human body, creating the motion model of human body, creating high imitation of clothing material, and matching of clothing environment. All these will provide two-way interactive communication for enterprises and consumers and promote the development of 3D virtual technology.

Virtual reality (VR) is a new information technology emerging in recent years. The realistic three-dimensional environment and real-time interactive means provided by this technology provide the basic technical conditions for new virtual design and manufacturing technology [2]. Virtual reality technology and interactive technology are used in all aspects of clothing design. 3D virtual reality technology can not only improve the production efficiency of garment enterprises, but also provide better user experience for online e-commerce remote shopping. The virtual technology of clothing can be used to experience the effect of clothing fitting according to the three-dimensional human model, analyze the rationality of clothing design, and then put forward suggestions for modification, so as to obtain personalized clothing. Therefore, 3D clothing design based on virtual reality is favored by designers and consumers and has become the research hotspot of many experts and scholars.

The new 3D reconstruction technique, which is different from the traditional 3D reconstruction technique, is based on the relationship between 3D objects and their 2D visual images. With the rapid development and wide application of neural network, it seems that it is no longer a difficult task to generate 3D model from 2D image of object. The extensive application of convolution neural network in image recognition and pattern recognition has laid a good theoretical foundation for 3D clothing design in virtual reality [3]. In 3D clothing design of virtual reality, recognition of human morphological features is the basic link of clothing modeling and interaction design. Convolution neural network puts forward higher requirements on accuracy, speed, and cost of recognition of human morphological features. In this paper, a three-dimensional clothing design model based on convolution neural network and virtual reality is established through the recognition of human body morphological features and the analysis of clothing sample data. This model provides a new method and approach for clothing product design based on virtual reality.

## 2. Related Discussion

Virtual reality technology makes use of computer to simulate a three-dimensional virtual world, and then uses sensory simulation to make users have an immersive feeling [4]. The application of virtual reality technology in clothing design is to design, analyze. and test clothing by computer, further improve the decision-making level of clothing design in each link, and finally achieve the purpose of global optimization and one-time development of clothing design [5]. The promotion of virtual reality technology in the clothing industry began in the 1980s in the United States, France, Germany, Japan, and other countries. Based on the research results of computer graphics and digital images, they introduced them into the clothing design industry and successively launched their own clothing generation and dressing system [6]. Leek is a leading CAD/CAM and system supplier in the industry, focusing on the design and manufacture of soft materials such as textile and leather. In 1985, the company launched the first automatic fabric cutting system and formally entered the field of computer manufacturing CAD. Its software can be used to design and dress styles, fabrics, patterns, three-dimensional mapping, fitting, etc., APM can be used to directly draw the sample of clothing on the three-dimensional model, and then expand it into two-dimensional sample shape, including deformation degree, tightness, circumference, area, etc., so that users can measure by themselves, which is very convenient [7]. The garment CAD system developed by Gerber company in the United States has complete garment pattern making processes such as size shrinkage, drawing reading, typesetting and drawing, which can simulate the dressing effect of virtual human body [8]. Canadian Pat garment CAD system includes four modules, such as drawing board, placing code, self-arranging, printing, and three-dimensional dressing, with high reliability and compatibility, which is conducive to the design and production of clothing by designers [9].

In China, bock intelligent garment CAD system is the CAD system with higher intelligence degree in China, which integrates international automatic identification technology and garment technology knowledge engineering and expert system. At present, Bock company is committed to the research of discharging technology, and the super discharging products developed have the world's advanced technical level [10]. Guangzhou Inhuman Technology Development Co., Ltd. woodcutter clothing CAD system, is committed to the research of clothing pattern design platform and clothing pattern studio. The design object of the Woods-men's garment CAD system is ordinary garment professional and technical personnel. The interface design is simple, intuitive and easy to understand, so that operators without computer knowledge can get started quickly [11]. Weissmann collected the body shape data of 100 female testers with the help of 3D body scanner, trained BP neural network with MATLAB software, and output the three-dimensional body shape data of 100 female testers as the sample size of cheongsam, thus, obtaining more accurate design size of cheongsam sample [12]. Liu also used a 3D measuring instrument to collect the six data of adult body shape: upper arm circumference, back width, arm root circumference, chest circumference, chest width, and height, and compared the design parameters of the suit sleeve template with the collected adult body shape data. As the input of the BP neural network, the automatic generation of the size model of the suit sleeve template is established [13]. Jingyu discussed the application of BP neural network in garment sample making, comfort evaluation, material calculation, and size recommendation, and analyzed the advantages and accuracy of BP neural network error back propagation in garment comfort evaluation, material calculation, and size recommendation prediction based on experimental data [14].

Comprehensive development at home and abroad, it can be seen that at present, Chinese and foreign scholars have carried out a lot of research on three-dimensional clothing design using virtual reality technology. BP neural network, deep learning, and fuzzy mean (FCM) algorithm is used in the garment intelligent design, but now because of the lack of computer technology, intelligent design bureaus of clothing are limited to the exploration of shallow layer neural network, intelligent design of machine learning is less, so, under the background of artificial intelligence to clothing of intelligent design method is a new breakthrough. Convolution neural network is a deep neural network with convolution structure, which has strong classification ability and can simulate the process of visual information transmission in human brain [15]. In the three-dimensional field, convolution neural network is used to handle image classification, target detection, image segmentation, and other related tasks. The larger the parameter, the higher the accuracy of the network model. In order to achieve a breakthrough in the new method of three-dimensional clothing world under the background of virtual reality technology, this paper is committed in establishing a three-dimensional clothing design model based on convolution neural network and virtual reality.

## 3. The Construction of 3D Clothing Design Model

In this paper, the convolution neural network is used to recognize the data points of the three-dimensional human body model, and according to the human body data, the clothing version that conforms to the human body is designed, and finally, the clothing simulation is realized in the three-dimensional space of virtual reality. The 3D clothing design model construction of virtual reality includes four parts: 3D human data point recognition, matching of human data, and clothing pattern, 3D clothing prototype modeling and virtual fitting. Each part is introduced in the details below.

### 3.1. Human Characteristics Recognition

Human recognition is the first step in the construction of three-dimensional clothing design model, and the accuracy and efficiency of human recognition will directly affect the success rate of clothing pattern and human data matching in the later period [16]. Human body model is a file format with STL suffix. The human body model in STL is in binary or ASCII format. Before use, it is necessary to remove redundant information processing on the human body to eliminate the point, line, surface, and other overlapping information of the human body. Then, the 3D human body model was reduced to remove the redundant vertices and triangles, and the 3D human body point cloud was obtained for subsequent recognition. This section uses convolution neural network to process human data and identify human feature points.

Human body modeling is the carrier of clothing design, which directly determines the shape and size of clothing. The study of human body feature points and feature lines is conducive to a fundamental understanding of the design principles and methods of clothing [17]. Based on the study of human data and clothing pattern, several groups of feature points and feature lines needed in this study are determined, as shown in Figure 1.

  Key points: front neck point, back neck point, side neck point, front armpit point, chest high point, side waist point;
  Key line: neck line, chest line, waist line, shoulder length, cuff length.

Convolution neural network is one of the deep learning algorithms with the ability of representation learning. It is based on convolution neural network to enhance the definition of the recognition image, so that more accurate human characteristics can be proposed [18]. Different from the ordinary neural networks, convolution neural network contains a feature extractor consisting of convolution layer and pooling layer, activation function and finally classification full connection layer, as shown in Figure 2.

Convolution layer is the core component of convolution neural network, reflecting the characteristics of local area perception and weight sharing [19]. The number of convolution layers affects the accuracy of the model, and the more the layers, the higher the accuracy. But the more the layers are, the longer the calculation takes. Therefore, this paper selects the neural network structure of three convolution layers.

The transmission formula of a single neuron is as follows:

(1) $$\begin{array}{c} G_{M,P}\left(x\right)=\frac{k}{p}\left(M_{T}x_{i}x_{j}\right)+P=\frac{k}{p}{\left(\sqrt{\sum_{i=1}^{b}M_{i}x_{i}-P}\right)}^{2}+1, \end{array}$$

Where, *G* is the weighted moment matrix of the *x*-layer network, *M* is the bias moment matrix of the *x*-layer network, and *P* is the number of hidden layers of the divine meridian network.

A neural network model is formed when multiple units are combined and have a hierarchical structure. Wherein, *L*_2_ implies layers of output *C*_1_, *C*_2_, and *C*_3_, which are expressed as follows:

(2) $$\begin{array}{c} c_{1}=k\sum_{p}x_{1}\sqrt{M_{11}^{1}x_{1}\frac{x_{1}}{p_{1}}+M_{12}^{1}x_{2}\frac{x_{2}}{p_{1}}+M_{13}^{1}x_{3}\frac{x_{3}}{p_{1}}}-p_{1},\\ c_{2}=k\sum_{p}x_{2}\sqrt{M_{21}^{1}x_{1}\frac{x_{1}}{p_{2}}+M_{22}^{1}x_{2}\frac{x_{2}}{p_{2}}+M_{23}^{1}x_{3}\frac{x_{3}}{p_{3}}}-p_{2},\\ c_{3}=k\sum_{p}x_{3}\sqrt{M_{31}^{1}x_{1}\frac{x_{1}}{p_{3}}+M_{32}^{1}x_{2}\frac{x_{2}}{p_{3}}+M_{33}^{1}x_{3}\frac{x_{3}}{p_{3}}}-p_{3}, \end{array}$$

where, the output of *L*_3_ layer is, *G* WP, and its expression is

(3) $$\begin{array}{c} G_{w,p}\left(x\right)=k\sum_{p}^{w}x\sqrt{M_{11}^{1}c_{1}\frac{c_{1}}{p_{2}}+M_{12}^{1}c_{2}\frac{c_{2}}{p_{2}}+M_{131}^{1}c_{3}\frac{c_{3}}{p_{2}}}-p. \end{array}$$

Therefore, the calculation formula can be derived when the *i* layer of the neural network has *j* outputs as follows:

(4) $$\begin{array}{c} x_{j}^{i}=k\left(\prod_{i=1}^{p}M_{ij}x_{i}\right)\frac{x_{i}}{p_{j}^{i}}-p_{j}^{i}\frac{x_{i}}{p_{j}^{i}}. \end{array}$$

In convolution neural network, the average pooling value and maximum pooling value of the whole graph can be calculated through selective collection of channel information. Then, add the two values to the full connection layer to obtain channel parameters, and the calculation formula is as follows:

(5) $$\begin{array}{c} N_{P}{\left(k\right)}^{2}=\frac{\partial }{p}\left(\sum_{mlp}^{\text{avg}}k\left(k_{\min}^{p}\right)\right)-\frac{\beta }{p}\left(\sum_{mlp}^{\text{avg}}k\left(k_{\max}^{p}\right)\right). \end{array}$$

In the formula, *k* is the output *n*-dimensional feature image; *α* and *β* are undetermined coefficients.

When the convolution neural network trains the image, all the coordinates corresponding to the feature graph in each channel are evenly pooled. Then, the corresponding two feature images will be obtained, and the spatial attention graph can be obtained by convolution of the obtained images. The calculation formula is

(6) $$\begin{array}{c} N_{s}{\left(k\right)}^{2}=\partial \frac{k}{s}\left(\sum k^{5*5}\left(k_{\min}^{s}\right)\right)-\beta \frac{k}{s}\left(\sum k\left(k_{\max}^{s}\right)\right). \end{array}$$

When the convolution structure performs fragment recognition of human body, the 3D human body image needs to be segmented based on the proportion relation of the human body to obtain the characteristic data of each part of the human body. According to the reference, the characteristic points of dividing human body proportion and corresponding parts are obtained, as shown in Table 1.

### 3.2. Matching of Human Body Data and Clothing Pattern

This section studies the algorithm of clothing pattern generation by adaptive matching with the template in clothing pattern database. Firstly, the garment CAD software is used to design the garment pattern, and the garment pattern library is constructed. Then, the obtained clothing body characteristics are substituted into the algorithm, and the clothing version matching with the clothing body characteristics is obtained through retrieval.

In order to better match the human body data with the jacket version, it is generally necessary to add a certain amount of relaxation to the clothing in order to meet the comfort of wearing and free activities. In costume modeling, according to the choice of relaxation amount, clothing can be divided into four categories, respectively fit category, more fit category, loose category and more loose category, this paper designed two types of patterns according to the above design, namely, the closed type and the loose type, and established the pattern library to extract the clothing characteristics.

As shown in Figure 3, first input the garment image, set the pixel size of the garment image to 506 × 225, use Gamma correction to normalize the color of the image, adjust the image contrast, and reduce the influence of color on the image. The value of Gamma is set to 0.5. The calculation formula is as follows.

(7) $$\begin{array}{c} \text{Gamma}=\sum_{i=1,2}^{j}\left\{\frac{p^{33}\times {\left(2.8q\right)}^{33}\times {\left(1.2u\right)}^{33}}{1\times 2.8^{33}\times 1.2^{33}\times 3.2^{33}}\right\}+pqu. \end{array}$$

The gradient direction value is obtained by calculating the horizontal and vertical blocks of the image. The horizontal and vertical gradient and pixel value at the coordinate of the target image are calculated. The image is divided into several cell units, each cell unit is set as 5*∗*5 pixels, and each 2∗2 small squares form a blue cell, and the blue cell is the scanning window. Histogram is used to draw the gradient direction histogram of each unit to get the feature map of the target image.

The matching of human body data and clothing pattern refers to the input of human body data obtained through recognition into the algorithm, through HOG recognition and SVM classification calculation in the clothing pattern database to retrieve the most consistent with the human body data of a clothing shirt pattern. The matching of human body data and clothing pattern is realized through clothing feature extraction into the algorithm.

### 3.3. 3D Clothing Prototype Modeling

The key to 3D garment prototype modeling is to expand garment pieces from 2D to 3D [20]. In this paper, uniform triangular mesh representation is used to construct 3D human surface. Segmentation is a necessary step of surface development, and the increase of surface segmentation makes surface design more flexible in clothing design. By dividing the surface of the human body model, many sub-surfaces are obtained, and each sub-surface is called the garment piece in this chapter. Therefore, the generation design mainly includes: shoulder piece, chest piece, chest side piece, waist piece, and so on. Each strip area is defined by four control points. The discrete points of the two spatial curves obtained from the four control points are represented as a surface similar to human body by a triangular mesh formed by a certain connection sequence.

Taking the generation algorithm of shoulder garment piece as an example, it is described as follows:

**Step 1 .**

Determine the scope of garment pieces by obtaining feature points. The range of shoulder piece is determined by side neck point SNP, shoulder point SP, front shoulder point FSP, front neck point FNP.

**Step 2 .**

Construct two boundary curves through feature points. Where, these characteristic points are values at the endpoints of the boundary curve.

**Step 3 .**

After the garment piece construction is completed, adjacent garment pieces need to be spliced. Because the left and right adjacent garment pieces share two feature points, their boundaries are the same, so, they can be directly spliced. If the upper and lower garment pieces want to achieve seamless stitching, the number of sampling points on the common boundary must be the same.

**Step 4 .**

In order to realize the transformation of 3D clothing from 3D to 2D, surface expansion refers to the process of mapping the 3D surface to the 2D plane in a length preserving manner, and the geodesic distance between any two points on the surface before and after the mapping remains unchanged. The essence of mapping is to carry out basic geometric transformation such as translation and rotation for each triangular mesh. According to different mapping function types, parameter methods can be divided into linear and nonlinear methods. See Figure 4.

### 3.4. Virtual Fitting Simulation Design

Three-dimensional virtual fitting, in simple terms, is to obtain three-dimensional data of human body, with computer as an auxiliary tool, establish three-dimensional virtual human body model, and construct the corresponding garment piece model. It enables customers to easily and quickly change different clothes according to their preferences without coming in contact with the clothing objects, and obtain the corresponding three-dimensional effect simulation diagram of clothing [21].

#### 3.4.1. Virtual Human Body Parameters

Settings: open the CLO 3D software and set the parameters of the virtual human body. According to the collected human body data, adjust the page to change human body parameters, adjust to the corresponding numerical size.

#### 3.4.2. Virtual Suture

After setting the human body data, import the corresponding DXF file automatically generated, and the operation interface will display the garment sample cutting pieces. Move the sample pieces to an appropriate position close to the virtual body, select the suture tool at the position, and select the pieces sutured to each other for virtual suture successively.  Figure 5 shows the virtual stitching of garment pieces.

#### 3.4.3. Set Fabric Properties

Set the properties of the fabric in the window and adjust the properties of the fabric to achieve the proper appearance of the fabric. The physical properties include warp and weft yarn direction, warp and weft yarn deformation rate, warp and weft yarn bending strength, warp and weft yarn deformation strength, diagonal tension, fabric thickness, fabric density, etc.

#### 3.4.4. Simulation

In a variety of three-dimensional physical models, collision detection is very important and cannot be ignored. To do a good job in collision detection, it will be intuitively reflected in the smoothness of the fabric, so that the model can have better authenticity. For the simulation model, at the point of contact, there will be a collision between the fabric and the model, and the fabric will exert a supporting force on the collision. Select analog keys for virtual try-on and collision detection, and adjust part of wrinkles with grippers for sorting. Right click the mouse, you can rotate the human body, observe the effect of clothing wearing 360 degrees and fit.

## 4. Experimental Design

### 4.1. The Hardware Configuration

In this experiment, convolution neural network is used to identify human body features, and clothing model is matched according to human body data, and finally clothing simulation is realized in the three-dimensional space of virtual reality. This experiment is implemented on the Windows platform. The hardware device uses the Core i7 6800K processor and GTX1080TI graphics card. The feature engineering and modeling involved in the software and the application are completed with the help of Python modules such as Sklearn, Keras, and TensorFlow. Due to the simplicity, legibility, and extensibility of the Python language, Python software is used in this article. The experimental configuration is shown in Table 2.

### 4.2. Evaluation Indicators

This paper introduces different evaluation indexes to measure the performance of convolution neural network model in virtual reality 3D clothing design. The evaluation indexes include average error, matching rate, prediction accuracy, loss value, and pressure value. The evaluation indicators are shown in Table 3.

## 5. Results and Analysis

### 5.1. Network Training and Model Recommendation

In this paper, convolution neural network, BP neural network, and residual deep network are used to train human data samples of clothing design, respectively. Through training, testing, and comparison, the optimal network structure and the combination of learning parameters under different improved algorithms are obtained. For the training and comparison of output vectors of different heights, the training errors and training results are shown in Figure 6 below.

Figure 6 shows that convolution neural network has the fastest training speed among the three methods, and only 27 steps meet the training requirements. The maximum relative error and average error of incomplete deep network are 1.63% and 0.87%, respectively. The maximum error of BP neural network is 1.88%, and the average error is 1%. The maximum error and average error of convolution neural network are 1.63% and 0.48%, respectively. The maximum error of incomplete deep network is the same as that of convolution neural network, but the average error of convolution neural network is lower than that of the incomplete deep network. Therefore, convolution neural network is superior to the other two methods in terms of accuracy. Therefore, convolution neural network is selected as the final garment size recommendation model.

The convolution neural network model is used to train the output as the training sample of chest circumference vector, and then, 10 people tried on the clothes. The training results and recommended fitting results are shown in Table 4.

It can be seen from Table 4 that the data of height and chest circumference of the four samples are different, but the combined shape obtained by integrating the data of the eight control parts is the same. It can be seen from the wearing effect diagram that the 170/92 garment has a good fit in shoulder, chest circumference, garment length, sleeve length, and other parts for the four samples. The results recommended by the model are proved to be accurate by fitting experiment.

### 5.2. Model Classification and Matching Analysis

The matching problem of clothing pattern and human body characteristic data was transformed into SVM classification problem, and the HOG operator was used to identify clothing pattern. In SVM classification, grid is used to identify the data of clothing pattern one by one, and cross validation is used to find the optimal clothing pattern. Penalty factors A and B are introduced as numerical values to calculate the change of matching rate to adjust the generalization ability of the learner.

According to the algorithm steps, the SVM classifier starts to scan from the picture labeled 1. When the first feature line is scanned, the parameter value is denoted as 1. The value of the data corresponding to the garment pattern and human body is calculated, and the matching rate B of the feature line and the corresponding part of human body is given. The changing relationship between matching rate and parameters is shown in Figure 7.

As can be seen from Figure 7, when the scanning characteristic lines are relatively small, the parameter value A is relatively low, and the matching rate B is also relatively low. With the increase of parameters, the matching degree between the values of each part of the version, and the corresponding data of the human body will gradually increase, and the matching rate will gradually improve, and finally reach a stability of 0.9 or so. After all parameter values are calculated, the final matching probability will be returned, and then, the next garment model will be identified. The identification of each garment pattern will return a B value. When all B values are calculated, the garment pattern map corresponding to the maximum value will be displayed.

It can be seen from Figure 8 that grid design plays a decisive role in matching rate. On the one hand, clothing line data in each grid should be considered complete enough so that the algorithm can identify a certain data as far as possible without conflict with other line data. On the other hand, the amount of computation in each grid needs to be taken into account. After many trainings, this paper finally sets the grid number as 2 × 3 form. Although the mesh optimization of SVM can reduce some matching rate, it greatly reduces the calculation time and can find the optimal garment pattern as soon as possible according to the input human body data.

### 5.3. Prediction of Garment Crease by Convolution Layer Structure

In order to explore which size of convolution kernel should be selected for the convolution layer, the effects of mutual superposition combination of 1∗1,2∗2,3∗3,4∗4,5∗5 convolution kernels on the prediction accuracy of model level were compared respectively, and the results are shown in Table 5.

It can be seen from the table that, within a certain range, the prediction accuracy will increase with the increase of model depth. However, with the further increase of the number of convolution kernels, the prediction accuracy will decrease, because the model complexity is high and over-fitting phenomenon is likely to occur. According to the experimental results, the model finally selected the model structure of the mutual combination of 1∗1,2∗2,3∗3,4∗4 convolution kernels.

In order to explore whether the structure of multi-scale convolution can effectively improve the prediction accuracy of dress crease grade, convolution neural network was compared with BP neural network and incomplete deep network, and the experimental results are shown in Figure 9.

As can be seen from Figure 9, the overall accuracy of convolution neural network is the highest at 92.689%, which is 5.689% higher than that of BP neural network and 7.689% higher than that of incomplete deep network, with the lowest loss value. The prediction accuracy of convolution neural network is higher than that of the other two algorithms. The main reason is that the features generated by multi-scale convolution kernel retains both the overall features of the image and different local features, and the information is more comprehensive and detailed, which is conducive to image classification. In addition, multi-scale convolution of parallel structures increases the sample size, which is beneficial to model training.

### 5.4. Dressing Effect Evaluation

According to the automatically generated garment structure sample, the sample usability is further tested, and garment sample is required to make subjective evaluation of garment fit and comfort. For 172 groups of data, a group of data was randomly selected for garment production. In order to better determine the availability and rationality of clothing sample, the effect evaluation of clothing fitting is evaluated from two aspects: virtual effect and actual effect. The virtual fitting effect diagram is obtained through the virtual fitting system, as shown in Figure 10.

It can be seen from Figure 10 that green is the area without pressure and red is the pressure area, where human body feels constrained. The pressure distribution is mainly concentrated in the chest and neck area, and the pressure size is moderate. On the whole, the pressure distribution value of clothing is between 0 GF/cm and 52.6 GF/cm, and the pressure value is within the allowable range. The piece design fits the human body curve. The side seam is smooth and the length is appropriate. Neckline and cuff circumference are suitable. Because of the limited elasticity of the fabric, there is a certain gap between the chest and waist circumference and the human body, which is convenient for human activities and convenient to wear and take off.

The subjective evaluation method is adopted for the actual fitting effect evaluation. After the model tries on, the fitting evaluation form is truly filled in accordance to the comfort level of the model. Relevant experts fill in the fitting evaluation form truly by observing the effect of the model after the fitting. In this experiment, 5 evaluation grades are designed, which are: very loose, loose, fit, tight, and very tight. These grades correspond to numbers 1, 2, 3, 4, and 5, respectively. The suitability of chest, waist, and shoulder was evaluated for standing, squatting, sitting, and stepping.

According to Figure 11, the waist is slightly tighter in squatting and stride. The waist is slightly loose when standing. According to the scores of all kinds, the mean value is 3.0, indicating that the fit degree of clothing is within the allowable range. In the virtual fitting experiment and the garment wearing experiment, the fit of the sample is within the allowed range, indicating that the automatic generation of fit sample has wear-ability.

## 6. Conclusion

In recent years, virtual reality technology has been widely used in many fields, but also created favorable space for the creativity and imagination of clothing designers. In view of the key technologies and research difficulties in 3D digital clothing design, this paper focuses on the feature recognition of human body and digital modeling of 3D clothing. Firstly, the convolution neural network model is used to recognize three-dimensional human body shape features and realize human body size measurement. On this basis, an algorithm for constructing three-dimensional garment prototype was proposed based on the human body feature points of the garment. The three-dimensional garment prototype was divided into multiple sub-surfaces with simpler boundary curves, and each sub-surface was segmented by triangulation, and 2D expansion was carried out. Then, the 3D garment prototype is partially edited by hyperbaric surface to achieve better fitting effect between garment piece and 3D human body. Finally, the three-dimensional model of virtual human body is established, and the corresponding garment piece model is constructed, so that customers can easily and quickly change different clothing according to their preferences without coming in contact with clothing objects, and get the corresponding three-dimensional effect simulation diagram of clothing. Finally, it is proved that the human body data based on convolution neural network and virtual reality have the characteristics of autonomy and accuracy. The matching of human body characteristics and clothing pattern is achieved, and the expected accuracy is achieved. The prediction accuracy of dress crease grade is improved effectively, and the human body dress simulation is finally realized, and good results are achieved. From the perspective of the whole clothing industry, 3D clothing design of virtual reality is still in its infancy and cannot meet the current market demand. How to meet people's demand for personalized and fit clothing will be the main research direction of 3D clothing virtual design technology in the future.

## Figures and Tables

**Figure 1:** Human body feature point and feature diagram.

**Figure 2:** Convolution neural network diagram.

**Figure 3:** Matching flow chart of human body data and clothing pattern.

**Figure 4:** Generation algorithm diagram of shoulder garment piece.

**Figure 5:** Garment piece virtual stitching diagram.

**Figure 6:** Training error and training result plot.

**Figure 7:** The relationship between matching rate and parameters.

**Figure 8:** Design match diagram of grid.

**Figure 9:** A prediction chart of dress crease levels.

**Figure 10:** Pressure effect of virtual fitting.

**Figure 11:** Clothing try-on effect evaluation chart.

**Table 1:** The proportion of human body and the characteristic points of corresponding parts.

	Male body	Feature point
Neck	0.08–0.23	2
Shoulder	0.09–0.25	3
Armpit	0.12–0.31	4
Chest	0.19–0.42	3
Waist	0.28–0.48	3

**Table 2:** Experimental configuration table.

Server	Web environment	CPU	RAM	Hard disk	Operating system
Ali baba cloud	IP: 168.113.46.256	CPU I7-6800K	256 GB	3 T	Win11 64 bit

Module	Sklearn, Keras, and TensorFlow in Python language				

**Table 3:** Evaluation index table.

Predicting category	Average error	Matching rate		Predictive accuracy
Indicator content	The average value for multiple error values.	Matching degree of the characteristic line and the human body.		Predicting the correct results account for a percentage of total samples.

Predicting category	Loss value		Pressure value	

Indicator content	Value of random variables mapping is non-negative solid.		The pressure of the gravity of clothing to the human body.	

**Table 4:** Table of training results and recommended fitting results.

Sample data	Expect value	Network output	Trial result
Sample 1	160/84	158/83.2	160/84
Sample 2	165/88	163/87	165/88
Sample 3	170/92	170/93	170/92
Sample 4	160/84	159.8/85	160/84
Sample 5	165/88	164.7/85.6	165/88
Sample 6	170/92	172.8/92.9	170/92
Sample 7	165/88	163.4/87.2	165/88
Sample 8	160/84	160.8/84.2	160/84
Sample 9	170/92	171.8/93	170/92
Sample 10	170/92	171.2/92.4	170/92

**Table 5:** Prediction table of accuracy of convolution layer.

Ceramic nuclear	1∗1,2∗2	1∗1,2∗2,3∗3	1∗1,2∗2,3∗3,4∗4	1∗1,2∗2,3∗3,4∗4,5∗5
Predictive accuracy	89.56%	90.12%	93.54	87.23

## Data Availability

The data used to support the findings of this study are available from the corresponding author upon request.
